# Analysis of Influencing Factors of Serum Stress Index and Prognosis of HICH Patients by Different Anesthesia Methods Combined with Small Bone Window Microsurgery

**DOI:** 10.1155/2022/6971092

**Published:** 2022-03-25

**Authors:** Guangping Zhao, Jiong Shi, Yongxue Chen

**Affiliations:** Anesthesiology Department, Handan Central Hospital, Handan 056001, China

## Abstract

In order to investigate the effects of sevoflurane on the serum stress index level and prognosis of patients with hypertensive cerebral hemorrhage (HICH) during small bone window microsurgery, a total of 102 HICH patients are selected for analysis. MAP values in both groups decreased significantly at T1 and T2 (*P* < 0.05), and the changes in MAP and HR indexes in the sevoflurane combined group were more stable than those in the control group. The time of postoperative awakening in the sevoflurane combined group decreases significantly than the control group (*P* < 0.001). The levels of T-AOC and GSH-Px in both groups increase significantly after operation, and those in the sevoflurane combined group increase significantly than the control group (*P* < 0.001). The levels of MDA and 8-OHDG in the sevoflurane combined group decrease significantly than the control group after operation (*P* < 0.05). Spearman correlation coefficient analysis shows that the levels of T-AOC and GSH-Px are negatively correlated with the prognosis of HICH patients, while MDA and 8-OHDG are positively correlated with the prognosis of HICH patients (*P* < 0.001). Sevoflurane interventional anesthesia has a high anesthetic effect in small bone window microsurgery, which has positive effects on controlling blood pressure of HICH patients, shortening postoperative recovery time and improving patients' stress response and neurological function. This paper conducts an in-depth analysis of the prognosis of HICH patients, indicating that the prognosis of HICH patients is closely related to their serum stress indicators T-AOC, GSH-Px, MDA, and 8-OHDG, providing a new direction for follow-up clinical diagnosis and treatment of HICH patients and accurate prognosis assessment.

## 1. Introduction

Hypertensive cerebral hemorrhage (HICH) is a common type of hypertension in severe complications; related data show that the incidence of HICH rise year by year. The onset of a ruptured blood vessel in the hindbrain resulting in cerebral hematoma and oppression of normal cells in the brain bring bad effects on the central nervous system. A series of pathophysiological reactions occur in patients with high risk of death and disability [1, 2]. Due to the rapid onset and progression of HICH, it is more difficult to improve and control the prognosis of HICH patients [3]. HICH patients progress in the process of the neural function damage, including primary and secondary damage. The former refers to patients with cerebral hemorrhage lesions caused by oppression brain tissue and nerve function damage after cerebral hemorrhage including primary and secondary damage; the process of the former pointed out that blood lesions in brain tissue compression was caused by the damage. The latter refers to damage caused by activation of oxidative stress response and increase of metabolites in the dynamic change of hematoma [4]. The main means of clinical treatment for cerebral hemorrhage is the removal of hematoma, combined with antioxidant drugs, which can relieve the oxidative stress response on the basis of the removal of bleeding focus and then reduce the primary and secondary damage of nerve function. At the present stage, the application of small bone window microsurgery can effectively remove the hematoma in the patient's brain and shorten the compression time of the hematoma on the brain tissue. The selection of effective anesthesia during the operation can effectively achieve the control of the patient's blood pressure and antihypertensive anesthesia. The reduction of side effects of anesthesia is conducive to faster recovery of patients and postoperative recovery of various functions, promoting the normal level of body indicators and improving prognosis [5]. Therefore, in this study, sevoflurane interventional anesthesia combined with minimally invasive surgery with a small bone window was analyzed to observe the effects of this operation on the serum stress index, neurological function index, and prognosis of HICH patients and further analyze the indicators affecting the prognosis of HICH patients.

The remainder of this paper is organized as follows: Section 2 presents the data and methods, and Section 3 provides the experimental results, followed by the result analysis inSection 4. Finally, the conclusions of this study and some future recommendations are given in Section 5.

## 2. Data and Methods

### 2.1. General Information

A total of 102 HICH patients admitted to our hospital from November 2020 to May 2021 were selected, and a sevoflurane combined group and control group were respectively established according to different anesthesia drugs, with 51 patients in each group. There were 33 males and 18 females in the sevoflurane combined group. The mean age was 59.12 ± 6.35 years ranging from 47 to 70 years. The course of hypertension ranged from 3 to 11 years, with an average of 6.76 ± 2.14 years. There were 26 cases of cerebral basal ganglia hemorrhage, 21 cases of cerebral lobe hemorrhage, and 4 cases of thalamic hemorrhage. According to HICH clinical classification criteria, 9 cases were grade I, 17 cases were grade II, 19 cases were grade III, and 6 cases were grade IV. According to the classification of the American Society of Anesthesiologists (ASA), 27 cases were grade II and 24 cases were grade III. In the control group, there were 36 males and 15 females, aged from 44 to 68 years, with a mean of 58.87 ± 6.64 years and 6.62 ± 2.05 years, respectively, and a course of hypertension of 2 to 10 years. There were 29 cases of hemorrhage at the basal ganglia, 20 cases of hemorrhage at the lobe, and 2 cases of thalamic hemorrhage. According to the evaluation of the clinical classification standard of hypertensive cerebral hemorrhage, 8 cases were grade I, 16 cases were grade II, 20 cases were grade III, and 7 cases were grade IV. All of them were grade II to III by the ASA grading assessment and 25 cases were grade II and 26 cases were grade III. There were no statistically significant differences in baseline data, such as gender, age, course of hypertension, site of cerebral hemorrhage, HICH clinical grade, and ASA grade between groups (all *P* > 0.05), which confirmed that the comparison between the groups was scientific and reasonable. Inclusion criteria were as follows: (1) imaging examination results and clinical manifestations of patients met HICH diagnostic criteria [6]; (2) it was evaluated by the Glasgow Coma Scale (GCS) with a score of 9–12 [7]; (3) the volume of supratentorial hematoma was ≥30 mL, and the volume of subtentorial hematoma was ≥10 mL; (4) no history of craniocerebral surgery; and (5) all patients had the first onset and the interval from onset to admission was less than 48 h. Exclusion criteria were as follows: (1) patients with severe liver, kidney, and other organic diseases or coagulopathy; (2) those with a history of mental illness or clinical manifestation of mental disorder; (3) patients with cerebral hemorrhage caused by cerebral aneurysm or trauma; and (4) patients with contraindications or allergic manifestations of the drugs used in this study.

### 2.2. Our Design Scheme and Method

#### 2.2.1. Anesthesia and Surgical Methods

Patients in both groups received anesthesia induction before surgery and received intravenous anesthesia. The drugs and corresponding doses were as follows: 0.05 mg/kg of midazolam (Jiangsu Nhwa Pharmaceutical Co. Ltd., H10980025, specification 2 mL:10 mg), fentanyl (Yichung Renfu Pharmaceutical Co. Ltd., H20003688, specification 10 mL:0.5 mg) 3 *μ*g/kg, propofol (Xi‘an Libon Pharmaceutical Co. Ltd., National drug approval H20010368, specification 10 mL:100 mg) 1.5 mg/kg, and vecuronium bromide (Chongqing Medicine you Pharmaceutical Co. Ltd., National drug approval H20084548, specification 4 mg) 0.1 mg/kg. After anesthesia induction, the control group received the following anesthesia maintenance regimen: the patients were pumped with propofol and remifentanil (produced by Yichung Renfu Pharmaceutical Co. Ltd., National drug approval H20030197, calculated as 1 mg C20H28N2O5). The Bispectral Index (BIS) was closely observed to ensure that it was maintained within the range of 40∼60. The sevoflurane combined group was treated with continuous inhalation of 1∼2% sevoflurane on the basis of an anesthesia maintenance program of the control group. After that, both groups received small bone window microincision. The specific steps were as follows: the incision was selected at the side of the mass closest to the cerebral cortex, the skin was opened with a spanner, the skull was exposed, the skull was expanded by drilling a hole to form a small bone window with a diameter of about 3 cm, and the dura was dissected in a cruciform. Under the microscope, part of the hematoma attached to the blood clot was repeatedly absorbed with a puncture needle. After no active bleeding, a drainage tube was indignant in the vascular cavity for drainage, the dura mater was sutured, and the brain was closed layer by layer. The intraoperative monitoring of intracranial pressure and drainage tube unobstructed will be done. After surgery, 20∼30 000 U urokinase was injected into the hematoma cavity. Drainage was performed 4∼6 hours later, and the drainage tube was removed when the hematoma volume was less than 10 mL. Propofol injection (1–4 mL/kg) was administered for sedation within 48 h after surgery, and the dosage was adjusted according to the patient's situation.

#### 2.2.2. Detection Method of Serum Indicators

5 mL of elbow venous blood in the fasting state was extracted 24 h and 7 d after surgery, and centrifuge operation was performed. The parameters were set to 3500 r/min, the centrifuge radius was 10 cm, and the duration was 10 min. Then, the supernatant was separated and an enzyme-linked immunosorbent assay was used to detect serum stress indicators, including total antioxidant capacity (T-AOC), malondialdehyde (MDA), 8-hydroxy glycoside (8-hydroxy-2) deoxyguanosine (8-OHDG), glutathione peroxidase (GSH-PX), neuron-specific enolase (NSE), neuropeptide Y(NPY), and brain-derived neurotrophic factor (BDNF). The kit was provided by Shanghai Jining Biological Co. Ltd. All indicators were tested strictly according to the kit instructions.

### 2.3. Observation Indicators

(1) Compare the differences of hemodynamic indexes between the two groups at different time periods; specifically mean arterial pressure (MAP) and heart rate (HR) before surgery (T0), before hypertensive arterial pressure (T1), 10 min after hypertensive arterial pressure (T2), and 40 min after hypertensive arterial pressure (T3) were observed. (2) The control time of hemodynamic indexes and postoperative recovery time were compared between the two groups. (3) The levels of serum stress indexes, including T-AOC, MDA, SOD, and GSH-Px, were compared between the two groups before and after surgery. (4) The levels of neurological function indexes, including NSE, NPY, and BDNF, were compared between the two groups. (5) The prognosis of the two groups was compared. (6) The Spearman correlation coefficient was used to analyze the correlation between the serum stress index level and the prognosis of HICH patients.

### 2.4. Criteria for Prognostic Assessment

The Glasgow Outcome Scale (GOS) was used for prognosis assessment 6 months after surgery [8]. Those with mild impairment of daily activities but normal daily life were judged to have recovered well. Those with mild disability, such as memory, language, and movement dysfunction, but independent in daily life can be assessed as moderate disability under the protection of workers. Persons with high mental and mobility impairments, poor independence, and the need for care in daily life are judged to be severely disabled. The patient developed vital signs after treatment, but was unconscious and lost language ability, which was determined as vegetative death. Excellent and good rate = (good recovery + moderate disability)/total number of cases × 100%.

### 2.5. Statistical Methods

This research collects the data and establishes the database. SPSS26.0 software was used for statistical analysis of measurement data to meet the normal distribution. The Mauchly test was used for data comparison. *P* > 0.05 indicated the symmetry of the covariance matrix. The Spearman correlation coefficient was used to analyze the correlation between the serum stress index level and prognosis of HICH patients, and *P* < 0.05 proved to be statistically significant.

## 3. The Experimental Results

### 3.1. Comparison of Hemodynamic Index Levels at Different Time Periods

There was no significant difference in the MAP index at T0 and T3 (*P* > 0.05). There was significant difference in the MAP index at T1 and T2, and the MAP value of the two groups decreased significantly at T2 (*P* < 0.05). There was no significant statistical difference in HR index levels at different time periods (*P* > 0.05). The changes in MAP and HR index levels in the sevoflurane combined group at different time periods were more stable than those in the control group.  Table 1 summarizes differences in MAP index levels at different time periods.  Table 2 shows differences in HR indicators between the two groups at different time periods.

### 3.2. The Control Time of Hemodynamic Indexes and Postoperative Recovery Time Were Compared

There were no significant differences in the time to reach the target MAP and the duration of controlled hypotension (all *P* > 0.05), but the time to wake up after operation in the sevoflurane combined group decreased significantly than that in the control group (*P* < 0.001).  Table 3 displays comparison of the control time of hemodynamic indexes, controlled hypotension time, and postoperative awakening time.

### 3.3. The Levels of Serum Stress Indexes Were Compared

Before surgery, there were no significant differences in T-AOC, MDA, 8-OHDG, and GSH-Px levels (all *P* > 0.05). The levels of T-AOC and GSH-Px in both groups increased significantly after operation, and the levels of indexes in the sevoflurane combined group increased significantly than the control group (*P* < 0.001). The levels of MDA and 8-OHDG indexes after surgery decreased significantly than those before the operation, and the indexes in the sevoflurane combined group decreased significantly than those in the control group (*P* < 0.05).  Table 4 shows comparison of serum stress index levels.

### 3.4. The Differences of Neurological Function Indexes

Before operation, there were no significant differences in NSE, NPY, and BDNF (all *P* > 0.05). After operation, the levels of NSE and NPY in the two groups decreased significantly, and the levels in the sevoflurane combined group decreased significantly than those in the control group (all *P* < 0.05). BDNF index levels in both groups increased significantly after operation, and comparison between the groups showed that the levels in the sevoflurane combined group increased significantly than those in the control group (*P* < 0.05), as shown in Table 5.

### 3.5. Comparison of Prognosis

Follow-up investigation is conducted 6 months after operation for patients in the two groups, which showed that the overall good and good rate of prognosis in the sevoflurane combined group increased significantly than that in the control group (*P* < 0.05), as shown in Table 6. The survival curve is shown in Figure 1.

### 3.6. The Correlation between the Serum Stress Index Level and Prognosis of HICH Patients Was Analyzed

Spearman correlation coefficient analysis shows that the levels of T-AOC and GSH-Px were negatively correlated with the prognosis of HICH patients, while the levels of MDA and 8-OHDG were positively correlated with the prognosis of HICH patients, with statistically significant differences (*P* < 0.001), as shown in Table 7.

## 4. The Experimental Analysis

Clinical manifestations of HICH are pupil narrowing, hematoma enlargement, complicated respiratory disturbance, and elevated blood pressure indicators [9]. Small bone window microincision interventional therapy can achieve rapid and accurate localization of the site of intracerebral hemorrhage in patients, and physicians can eliminate intracerebral hematoma in a short time, thus reducing the risk of postoperative complications [10]. However, the intraoperative anesthesia method and its effect on patients are also important factors affecting the success rate of surgery. If the intraoperative anesthesia effect is not good, it may cause irreversible damage to the body of HICH patients and adversely affect their postoperative recovery [5]. It should be noted that HICH disease mostly occurs in middle-aged and elderly people, so anesthetic drugs with little influence on the patient's body should be selected before surgical treatment to ensure the safety and effectiveness of the whole surgical treatment [11]. Sevoflurane is a new type of halogen anesthetic, which has been applied to surgical anesthesia with an obvious anesthetic effect. Compared with inhalation anesthetic drugs previously applied in clinical practice, sevoflurane has less irritation to the patient's respiratory tract, rapid induction of anesthesia, and is nontoxici [12]. At present, some scholars have observed the anesthetic effect of sevoflurane in craniotomy on patients with craniocerebral injury and found that the drug can effectively reduce the degree of nerve injury in patients [13]. However, no scholars have applied sevoflurane in small bone window microincision, and the effects of this drug on stress response, neurological function, and prognosis of HICH patients have not been reported.

In this study, there were significant differences in MAP and HR levels before and after hypotension in each group *P* < 0.05From the point of change trend, sevoflurane joint group changes more smoothly, and the group of postoperative revival is significantly shortened than the control group *P* < 0.05. As a kind of volatile anesthetics, sevoflurane can act directly on the nervous system and then affect the hemodynamics of patients. Other results showed that sevoflurane had no significant effect on excitatory amino acids and dopamine, but when patients were in a state of continuous ischemia, sevoflurane intervention had a certain inhibitory effect on the increase of excitatory amino acids and dopamine levels and actively acted on the renin-angiotensin system, so as to increase cerebral blood flow and increase the blood supply of brain tissue. In addition, it is beneficial to maintain the integrity of blood vessel wall and the blood internal environment and reduce and protect the ischemic damage of brain tissue [14]. This study also fully confirmed that sevoflurane interventional anesthesia has high safety.

In order to further explore the effects of sevoflurane on HICH patients, this study conducted a comparative analysis of the changes of serum stress indicators and neurological function indicators in the two groups, showing that all indicators were significantly improved in the sevoflurane combined group. It should be noted that HICH patients are prone to stress response after onset, which is also a secondary case factor of further aggravation of brain injury in patients. Stress response of patients causes massive proliferation of various cytokines, which is an important mechanism of aggravating brain edema and impaired brain function [15]. Studies have pointed out that MDA is a marker of lipid oxidative damage and the level of this indicator is closely related to the early onset and severity of HICH [16]. 8-OHDG is an oxidative adduct and a marker of oxidative damage to DNA caused by endogenous and exogenous factors [17]. GSH-Px is an important peroxide decomposition enzyme widely existing in the body, which reduces toxic peroxides to nontoxic hydroxyl compounds, so as to protect the structure and function of cell membranes from interference and damage by oxides [18]. In combination with the changes of oxidative stress indexes, HICH patients had a high degree of oxidative stress response in serum, and a high degree of oxidative stress response would damage the neurological function of patients. Restoration of cerebral blood supply is the material basis for the protection of nerve cells. When cerebral ischemia occurs, a large number of factors such as NSE and NPY are released into the blood through the damaged membrane, so the high level of NSE and NPY in serum is a sign of brain injury, and the level of NSE and NPY is consistent with the severity of brain injury [19, 20]. BDNF is a protein with neurotrophic effects, which is widely distributed in the nervous system. Existing studies have shown that when nerve injury occurs, the generation and release of BDNF is impaired, which further leads to irreversible apoptosis of nerve cells [21].

This study compared the prognosis of the two groups 6 months after surgery and showed that the good and good prognosis rate of sevoflurane combined group was significantly higher than that of the control group. In order to further explore the influencing mechanism of prognosis of HICH patients, the Spearman correlation coefficient was used to analyze the correlation between the serum oxidation index and the prognosis of patients. It was found that the levels of T-AOC, MDA, SOD, and GSH-Px were closely correlated with the prognosis of patients, which may be because oxidative stress is one of the basic mechanisms of oxidative damage of brain tissue during intracerebral hemorrhage. Oxidative stress reaction is involved in the pathological process of brain tissue damage in patients with intracerebral hemorrhage. A large number of oxygen-free radicals are formed in the lesion area, exacerbating nerve cell damage in the area around the lesion. Meanwhile, related oxygen-free radicals can also pass through the blood-brain barrier and cause systemic oxidative stress injury, leading to poor prognosis of patients [22–24]. This finding also provides new ideas for accurate follow-up clinical assessment of patients' prognosis and further confirms that sevoflurane interventional surgical anesthesia can inhibit patients' oxidative stress state and play an important role in improving patients' prognosis [25, 26].

The sample size and sample selection in this study is less, postoperative follow-up work time is shorter than the deficiency existing in this research, and current clinical trials is less related to this study.A follow-up study should expand the sample size and sample range and select multiple follow-up time points. This paper compares and analyzes of HICH conditions for the further study of the impact mechanism, to provide more reference data for improving the curative effect and prognosis of HICH surgery.

## 5. Conclusion

The anesthetic effect of sevoflurane intervention is more obvious for HICH patients in small bone window microsurgery, and its clinical application has high safety. It can reduce patients' stress response, cause little damage to nerve function, and also promote the improvement of prognosis, which is worthy of clinical application. In addition, this study further analyzed the prognostic mechanism of HICH patients and found that serum stress indicators are closely related to patients' prognosis, suggesting that follow-up clinical improvement of HICH patients' diagnosis and treatment plan can start from the control of patients' stress indicators, providing a new direction for further improvement of patients' prognosis.

## Figures and Tables

**Figure 1:** Survival function at 6 months after surgery.

**Table 1:** Differences in MAP index levels at different time periods (mmHg, ‾*x* *±* *s*).

Group	T0	T1	T2	T3

Sevoflurane combined group (*n* = 51)	91.86 ± 8.42	89.03 ± 7.85	77.32 ± 5.24^#^	88.79 ± 7.92^△^
Control group (*n* = 51)	92.14 ± 8.57	101.47 ± 8.53^*∗*^	74.56 ± 5.31^*∗*#^	89.64 ± 7.83^#△^
*t*	−0.761	−7.664	2.642	−0.545
*P*	0.449	<0.001	0.010	0.587
Between groups	*F* = 4.672, *P*=0.000			
Different points in time	*F* = 4.154, *P*=0.000			
Between groups · different time points	*F* = 3.741, *P*=0.000			

*Note.* ^*∗*^ represents *P* < 0.05 compared with T0; ^#^ represents *P* < 0.05 compared with T1; and ^△^ represents *P* < 0.05 compared with T2.

**Table 2:** Differences in HR indicators between the two groups at different time periods (times/min, ‾*x* *±* *s*).

Group	T0	T1	T2	T3

Sevoflurane combined group (*n* = 51)	81.46 ± 7.63	79.25 ± 7.34	71.72 ± 6.56^*∗*#^	80.86 ± 7.28^△^
Control group (*n* = 51)	80.82 ± 7.57	77.57 ± 7.21^*∗*^	72.44 ± 6.78^*∗*#^	81.42 ± 7.04^#△^
*t*	0.425	1.166	−0.545	−0.395
*P*	0.672	0.246	0.587	0.694
Between groups	*F* = 5.151, *P*=0.000			
Different points in time	*F* = 5.235, *P*=0.000			
Between groups · different time points	*F* = 4.526, *P*=0.000			

*Note.* ^*∗*^ represents *P* < 0.05 compared with T0; ^#^ represents *P* < 0.05 compared with T1; and ^△^ represents *P* < 0.05 compared with T2.

**Table 3:** Comparison of the control time of hemodynamic indexes, controlled hypotension time, and postoperative awakening time (min, ‾*x* *±* *s*).

Group	Time to reach the target MAP	Controlled hypotension time	Waking up after surgery

Sevoflurane combined group (*n* = 51)	10.87 ± 2.64	40.78 ± 8.76	5.17 ± 1.15
Control group (*n* = 51)	11.16 ± 2.75	38.25 ± 8.03	8.72 ± 1.64
*t*	−0.543	1.520	−12.657
*P*	0.588	0.132	<0.001

**Table 4:** Comparison of serum stress index levels (‾*x* *±* *s*).

Group	T-AOC (U/L)		MDA (nmol/L)		8-OHDG (*μ*g/L)		GSH-Px (U/L)	
	Before operation	After operation	Before operation	After operation	Before operation	After operation	Before operation	After operation

Sevoflurane combined group (*n* = 51)	0.96 ± 0.08	3.26 ± 0.24^*∗*^	3.85 ± 0.31	2.17 ± 0.18^*∗*^	9.18 ± 0.85	4.65 ± 0.52^*∗*^	87.26 ± 8.79	175.92 ± 16.06^*∗*^
Control group (*n* = 51)	0.94 ± 0.07	2.52 ± 0.15^*∗*^	3.91 ± 0.34	2.59 ± 0.22^*∗*^	9.47 ± 0.93	5.54 ± 0.68^*∗*^	86.75 ± 8.64	148.63 ± 14.33^*∗*^
*t*	1.344	18.672	−0.931	−10.522	−1.644	−7.425	0.295	9.055
*P*	0.182	<0.001	0.354	<0.001	0.103	<0.001	0.768	<0.001

*Note.* ^*∗*^ represents comparison with before the operation. *P* < 0.05

**Table 5:** Comparison of neurological function indexes (‾*x* *±* *s*).

Group	NSE (mg/L)		NPY (ng/L)		BDNF (ng/mL)	
	Before operation	After operation	Before operation	After operation	Before operation	After operation

Sevoflurane combined group (*n* = 51)	22.86 ± 2.84	10.27 ± 1.13^*∗*^	232.41 ± 20.86	125.64 ± 12.78^*∗*^	4.12 ± 0.68	7.47 ± 0.94
Control group (*n* = 51)	23.14 ± 2.92	14.35 ± 1.36^*∗*^	234.62 ± 21.11	141.86 ± 13.05^*∗*^	4.03 ± 0.61	5.14 ± 0.77
*t*	−0.491	−16.478	−0.532	−6.381	0.704	13.694
*P*	0.625	<0.001	0.596	<0.001	0.483	<0.001

*Note.* ^*∗*^ represents comparison with before the operation, *P* < 0.05.

**Table 6:** Comparison of prognosis 6 months after operation (*n*, %).

Group	Good recovery	Moderate disability	Severe disability	Plant response	Death	Excellent

Sevoflurane combined group (*n* = 51)	22 (43.14)	16 (31.37)	4 (7.84)	4 (7.84)	5 (9.80)	38 (74.51)
Control group (*n* = 51)	13 (25.49)	14 (27.45)	6 (13.73)	5 (9.80)	13 (25.49)	27 (52.94)
*x* ^2^	—	—	—	—	—	5.132
*P*	—	—	—	—	—	0.023

**Table 7:** Correlation analysis of serum stress indexes and prognosis of HICH patients.

Indicators	Poor prognosis	
	*rs*	*P*

T-AOC	−0.655	<0.001
MDA	0.707	<0.001
8-OHDG	0.650	<0.001
GSH-Px	−0.654	<0.001

## Data Availability

The simulation experiment data used to support the findings of this study are available from the corresponding author upon request.
